The article "Prevalence and associations of depression, anxiety, and stress among people living with HIV: A hospital‐based analytical cross‐sectional study" was published in 2022. Journal: Health Sci Rep.

# Prevalence and associations of depression, anxiety, and stress among people living with HIV: A hospital‐based analytical cross‐sectional study

**DOI:** 10.1002/hsr2.754

**Published:** 2022-08-08

**Authors:** Sampson Opoku Agyemang, Jerry Ninonni, Lydia Bennin, Elizabeth Agyare, Leveana Gyimah, Kafui Senya, Emmanuel Birikorang, Emmanuel Nii‐Boye Quarshie, Nyonuku Akosua Baddoo, Stephen Ayisi Addo, Dorcas Obiri‐Yeboah

**Affiliations:** ^1^ Department of Mental Health, School of Nursing and Midwifery University of Cape Coast Cape Coast Ghana; ^2^ Public Health Unit, Cape Coast Teaching Hospital Cape Coast Ghana; ^3^ Communicable and Non‐Communicable Diseases Cluster World Health Organisation Country Office Accra Ghana; ^4^ Department of Laboratory Technology, School of Physical Sciences University of Cape Coast Cape Coast Ghana; ^5^ Department of Psychology, School of Social Sciences University of Ghana Accra Ghana; ^6^ National AIDS/STIs Control Programme Accra Ghana; ^7^ Department of Microbiology and Immunology, School of Medical Sciences University of Cape Coast Cape Coast Ghana

**Keywords:** anxiety, depression, Ghana, mental health, people living with HIV, stress

## Abstract

**Background and Aims:**

An important but much less researched burden of human immunodeficiency virus (HIV) in Sub‐Saharan Africa includes the associated mental health outcomes of living with the virus. This study aimed to estimate the prevalence of depression, anxiety, and stress, and describe some of the socio‐demographic associations among people living with HIV (PLHIV) in Ghana.

**Methods:**

A cross‐sectional study was conducted at the Cape Coast Teaching Hospital, Ghana. Simple random sampling was used to recruit 395 PLHIV who access HIV‐related services at the antiretroviral therapy clinic. The Depression, Anxiety, and Stress Scale‐21 was used to assess prevalence of depression, anxiety, and stress. Frequencies and percentages were used to estimate the prevalence and multivariable logistic regression was used to evaluate sociodemographic factors associated with depression, anxiety, and stress.

**Results:**

The prevalence estimates of depression, anxiety, and stress among PLHIV were 28.6% (95% confidence interval [CI] 24.4–33.3), 40.8% (95% CI = 36.0–45.8), and 10.6% (95% CI = 7.9–14.1), respectively. Females reported higher prevalence of depression (32.2%; 95% CI = 27.2–37.7), anxiety (44.0%; 95% CI = 38.4–49.6), and stress (12.6%; 95% CI = 9.4–17.0) compared to depression (17.5%; 95% CI = 11.1–26.4), anxiety (30.9%; 95% CI = 22.5–40.7), and stress (4.1%; 95% CI = 1.2–10.4) among males. PLHIV without a regular partner were about 0.63 increased odds of experiencing anxiety compared to those with a regular partner (AOR = 0.63, 95% CI = 0.40–1.00: *p* = 0.049). PLHIV without formal education were about 0.49 and 0.44 increased odds to experience anxiety and stress, respectively compared to those with tertiary education.

The article "Prevalence and associations of depression, anxiety, and stress among people living with HIV: A hospital‐based analytical cross‐sectional study" was published in 2022. Journal: Health Sci Rep.

**Conclusions:**

Generally, the levels of stress, anxiety, and depression are high among PLHIV, but disproportionately higher among females. Mental health assessment and management should be integrated into the HIV care services. There should be capacity building for health care workers to offer differentiated service delivery based on mental health care needs of PLHIV.

## 1 BACKGROUND

Human immunodeficiency virus/acquired immunodeficiency syndrome (HIV/AIDS) remains a global menace and impacts significantly on the lives of individuals and their families despite the significant advances in its prevention and treatment. It is claimed that full gains of prevention and treatment will not be achieved without addressing the mental health needs of people living with HIV (PLHIV).^1^ In Ghana, it is estimated that there are about 342,307 people (122,321 males and 219,986 females) living with HIV, representing a 12‐month prevalence rate of about 2%.^2^ The chronicity of HIV/AIDS is not only impacting on physical health but is also having enormous challenges on psychological wellbeing.^3^ In particular, HIV‐related stigma, depression, anxiety, and stress have been reported among PLHIV.^4^, ^5^, ^6^

Thus, a major burden of living with HIV relates to the negative mental health outcomes and the psychosocial impact of the disease, including stigma, depression, anxiety, self‐esteem, loneliness, and reduced quality of life.^3^, ^4^ Studies suggest that PLHIV often suffer from depression and anxiety disorders as they adjust to the diagnosis, struggle with the meaning of a positive test result, adapt to life with chronic, life‐threatening illness, and witness of the death of a family member or a friend with HIV/AIDS.^7^, ^8^

Evidence suggests higher estimates of mental disorders in PLHIV. Recent studies from high‐income countries, for example, the United States, suggest a 36% prevalence of depression and 16% anxiety disorders among a large national sample of HIV‐positive men and women during the previous 12 months.^9^ In sub‐Sahara Africa, the prevalence of mental disorders among PLHIV during a period of 3 months was estimated to be as high as 19%.^10^ For example, it is estimated that 32% and 34.4% of people living with HIV in South Ethiopia suffer from depression and anxiety, respectively.^4^

Given the evidence of strong association of poor mental health outcomes with living with HIV, there is a need for both targeted and universal mental health screening and having mental health prevention and treatment options integrated into HIV care regimes.^1^ Although mental health has been integrated into the care of HIV/AIDS mostly in high‐income countries as a result of substantial evidence supporting the linkage between mental health and HIV, little is still known in sub‐Sahara African countries, including Ghana.^8^

The article "Prevalence and associations of depression, anxiety, and stress among people living with HIV: A hospital‐based analytical cross‐sectional study" was published in 2022. Journal: Health Sci Rep.

Considering that Ghana is a signatory to the UN 2030 Agenda for Sustainable Development, we believe a carefully designed study like the current one can, potentially, contribute evidence that supports the country's broad efforts towards attaining Goal 3 of the Sustainable Development Agenda: “Ensuring healthy lives and promote well‐being for all at all ages.”^11^ Specifically, this study sought to estimate the prevalence of mental health challenges and describe some of the socio‐demographic associations among PLHIV presenting to a teaching hospital in Ghana. This paper focuses on the prevalence and factors associated with depression, anxiety, and stress.

## 2 METHODS

### 2.1 Study design and study area

This is a hospital‐based analytical cross‐sectional study conducted at the Cape Coast Teaching Hospital in Ghana, between May and December 2021. The hospital has the highest number of clients at the antiretroviral therapy (ART) clinic in the Central Region of Ghana. It is a 400‐bed capacity teaching hospital affiliated with the School of Medical Sciences at the University of Cape Coast, Ghana.

## 3 POPULATION AND SAMPLING PROCEDURE

The population for this study included all adults (aged 18 years and above) living with HIV/AIDS who received service from the Cape Coast Teaching Hospital. Data available from the facility in the year 2019 suggested that there were 3972 PLHIV presenting to the facility. The inclusion criteria for this study were adults aged at least 18 years with a confirmed diagnosis of HIV/AIDS for at least 12 months and receiving care at the Cape Coast Teaching Hospital. The first 6 months of ART are critical in the care of PLHIV. Some PLHIV may not respond as expected to the treatment or may even deteriorate clinically.^3^ This would have affected the findings of this study. Therefore, people living with HIV on ART for 12 months were considered eligible for this study.

The sample size was predetermined by applying the Miller and Brewer's formula: at 95% confidence level, *n* = $\frac{N}{\left(1+N{\left(a\right)}^{2}\right)}$. Where: *n*= desired sample size, *N* = target population (3972), *a* = level of statistical significance (0.05), and 1 is a constant.^12^

Therefore, *n* (the predetermined sample size) = 363. However, to make up for incomplete data, the sample size was increased by 10% bringing the predetermined sample size to 399.^13^

The article "Prevalence and associations of depression, anxiety, and stress among people living with HIV: A hospital‐based analytical cross‐sectional study" was published in 2022. Journal: Health Sci Rep.

A simple random sampling technique was used to recruit participants. The sample frame was determined by acquiring the list of all adults living with HIV/AIDS who received service from the ART clinic from the hospital's records department. Each name in the sample frame was numbered. A random number generator was used to generate random numbers and registered the name in the sample frame corresponding to the numbers to constitute the sample. This was continued until the required number of participants (399) was met.

## 4 MEASURES

Data were collected using a self‐report anonymous questionnaire. The questionnaire had three sections. The first section focused on socio‐demographic characteristics of participants (e.g., age, gender, education, marital status, employment status, information on antiretroviral medication, other underlying physical health conditions, and support networks). The final section of the questionnaire comprised the Depression, Anxiety and Stress Scale‐21 (DASS‐21)—a set of three self‐report scales designed to measure the states of depression, anxiety, and stress among adults.^14^ Each of the three DASS‐21 subscales contains seven items with similar contents. DASS‐21 is a 21‐item self‐report scale on a 4‐point scale: 0—(did not apply to me at all—never), 1—(applied to me some of the time—sometimes), 2—(applied to me a considerable degree—often), and 3—(applied to me most of the time—almost always). Some example items are “I found it hard to wind down,” “I experienced trembling,” I felt down‐hearted and blue.” Participants indicated how much a statement applied to them over the previous 1 week. Scores for depression, anxiety, and stress were calculated by summing the scores for the relevant items: depression (normal = 0–4, mild = 5–6, moderate = 7–10, severe = 11–13, and extremely severe = 14+), anxiety (normal = 0–3, mild = 4–5, moderate = 6–7, severe = 8–9, and extremely severe = 14+), and stress (normal = 0–7, mild = 8–9, moderate = 10–12, severe = 13–16, extremely severe = 17+). DASS‐21 has satisfactory Cronbach alpha for each subscale (depression = 0.88, anxiety = 0.82, and stress = 0.90).^15^

Five research assistants with at least a bachelor's degree were recruited to assist with data collection. They were trained on the type of information to be collected from participants and how to uphold the ethical position of the data collection process and the entire study protocol. The training lasted for 4 h and ensures that they understood the data collection instrument. The questionnaires were administered privately to each participant by the first author or a trained research assistant at a convenient place at the ART clinic (e.g., selected consulting rooms). Averagely, it took each participant approximately 20 min to complete the questionnaire. Participants who were not literate were assisted by the first author or research assistants to complete the questionnaire. Three hundred and ninety‐five questionnaires were returned with complete data, yielding a response rate of 99%.

The article "Prevalence and associations of depression, anxiety, and stress among people living with HIV: A hospital‐based analytical cross‐sectional study" was published in 2022. Journal: Health Sci Rep.

Pre‐testing of the instrument was conducted to establish the appropriateness of the instrument and determine how feasible they would translate into the local dialect in the full‐scale study. The instrument was administered to 40 people and the feedback from pretesting was used to improve the use of the instrument.

This study was performed in accordance with the Helsinki Declaration and approved by the Ethics Review Committee of Cape Coast Teaching Hospital, Ghana (reference: CCTHERC/EC/2021/028). The purpose of the study, anonymity, voluntary participation, and confidentiality of the information were explained to participants to seek their written consent. Only those who gave written informed consent were included in the study. Participants could withdraw from the study at any point without any adverse effect. The hospital where the study was carried out gave permission for the study to be carried out.

## 5 DATA ANALYSIS

STATA version 16 was used for the statistical analysis. Frequencies and percentages were used to estimate the prevalence, summary statistics was based on the distribution of the data. For normally distributed variables, mean and standard deviation was used. Bivariable analysis using *t‐*test or *χ* ^2^ test (as appropriate) and multivariable logistic regression were used to evaluate sociodemographic factors and risky health behaviors associated with depression, anxiety, and stress. Age and gender were the only a priory variable. Sociodemographic variables were included in the final logistics model regardless of the statistical significance of their bivariable associations with the outcomes. However, variables with acute sparse data were excluded.^16^ For ease of data interpretation, each of the outcomes (depression, anxiety, and stress) were dichotomized. The response categories “mild,” “moderate,” “severe,” and “extremely severe” were merged and renamed “depressed,” “anxious,” and “stressed,” while the remaining response category, “normal,” was maintained to indicate “normal mood level,” “normal anxiety level,” and “normal stress level.” Statistical significance was based on the *p*‐value (*p* < 0.05) and associated 95% confidence interval (95% CI).

## 6 RESULTS

### 6.1 Demographic data of participants

Out of 395 participants recruited for this study, 52.2% (*n* = 206) were within the 40–59 years group (mean: 46.79; SD: ±12.53), and 75.4% (*n* = 298) of the participants were female. It was found that 61.8% (*n* = 244) of the participants were without a regular partner and 16.7% (*n* = 66) reported having additional comorbidities. Additionally, 77.7% (*n* = 307) of the participants were self‐employed (Table 1).

The article "Prevalence and associations of depression, anxiety, and stress among people living with HIV: A hospital‐based analytical cross‐sectional study" was published in 2022. Journal: Health Sci Rep.

**Table 1:** Socio‐demographic and clinical characteristics of participants (*N* = 395)

Characteristic	Category	*n* (% or SD)
Age (years)		
	Mean	46.7 (12.5)
	20–39	122 (30.8)
	40–59	206 (52.2)
	60–80	67 (17.0)
Gender		
	Male	97 (24.6)
	Female	298 (75.4)
Marital status		
	Currently with a regular partner	151 (38.2)
	Currently without a regular partner	244 (61.8)
Religion		
	Christian	355 (89.9)
	Islam	31 (7.8)
	Traditionalist	3 (0.8)
	No religion	6 (1.5)
Employment status		
	Employed by other	12 (3.0)
	Employed by self	307 (77.7)
	Unemployed	76 (19.2)
Educational level		
	Tertiary	38 (9.6)
	Nontertiary	246 (62.3)
	No education	111 (28.1)
Do you drink alcohol?		
	Yes	17 (4.3)
	No	378 (95.7)
Have a comorbid condition(s)		
	Yes	66 (16.7)
	No	329(3.3)

The topmost co‐morbid conditions were hypertension (60.6%, *n* = 40) followed by diabetes (7.6%, *n* = 5) and asthma (6.1%, *n* = 4) (Figure 1).

**Figure 1:** Prevalence of comorbid health conditions among participants (*N* = 66). “Other conditions” included peptic ulcer and uterine fibroids.

### 6.2 Prevalence estimates of depression, anxiety, and stress

Overall, varying prevalence estimates of depression (8.6%; 95% CI = 24.4–33.3), anxiety (40.8%; 95% CI = 36.0–45.8), and stress (10.6%; 95% CI = 7.9–14.1) were reported during the past week among PLHIV. As shown in Table 2, notably, relative to males, higher estimates were reported among females across the three outcomes.

**Table 2:** Prevalence estimates of depression, anxiety, and stress among participants (*N* = 395)

Characteristics	Variables					
	Depression		Anxiety		Stress	
	*n* (%)	95% CI	*n* (%)	95% CI	*n* (%)	95% CI
Overall	113 (28.6)	24.4–33.3	161 (40.8)	36.0–45.8	42 (10.6)	7.9–14.1
Female	96 (32.2)	27.2–37.7	131 (44.0)	38.4–49.6	37 (12.4)	9.4–17.0
Male	17 (17.5)	11.1–26.4	30 (30.9)	22.5–40.7	4 (4.1)	1.2–10.4

Abbreviation: CI, confidence interval.

## 7 FACTORS ASSOCIATED WITH DEPRESSION, ANXIETY, AND STRESS

### 7.1 Depression

Overall, only gender showed a statistically significant independent association with depression. Specifically, the multivariable logistic analysis (Table 3) showed that females were at approximately 0.5 increased odds of experiencing depression during the previous week compared to males (AOR = 0.48, 95% CI = 0.25–0.91: *p* = 0.03).

The article "Prevalence and associations of depression, anxiety, and stress among people living with HIV: A hospital‐based analytical cross‐sectional study" was published in 2022. Journal: Health Sci Rep.

**Table 3:** Factors associated with depression, anxiety, and stress

Characteristics	Depression			Anxiety			Stress		
	*χ* ^2^ (*p*)	AOR (95% CI)	*p*	*χ* ^2^ (*p*)	AOR (95% CI)	*p*	*χ* ^2^ (*p*)	AOR (95% CI)	*p*
*Age*	*1.16 (0.56)*	*‐*	*‐*	*1.04 (0.59)*	*‐*	*‐*	*1.97 (0.37)*	*‐*	*‐*
20–39	‐	Ref	‐	‐	Ref	‐	‐	Ref	‐
40–59	‐	1.23 (0.59–2.58)	0.58	‐	1.65 (0.85–3.21)	0.14	‐	0.63 (0.21–1.84)	0.39
60–80	‐	1.38 (0.70–2.66)	0.36	‐	1.35 (0.74–2.47)	0.33	‐	0.87 (0.35–2.17)	0.77
*Gender*	‐	‐	‐	‐	‐	‐	‐	‐	‐
Male	7.73 (0.003)	Ref	‐	5.15 (0.02)	Ref	‐	5.73 (0.01)	Ref	‐
Female	‐	0.48 (0.25–0.91)	0.03	‐	0.78 (0.45–1.34)	0.36	‐	0.34 (0.11–1.04)	0.06
*Marital status*	*1.42 (0.14)*	*‐*	*‐*	*5.92 (0.01)*	*‐*	*‐*	*0.43 (0.31)*	*‐*	*‐*
Currently with a regular partner	‐	Ref	‐	‐	Ref	‐	‐	Ref	‐
Currently without a regular partner	‐	0.87 (0.53–1.42)	0.56	‐	0.63 (0.40–1.00)	0.05	‐	1.81 (0.89–3.69)	0.10
*Religion*	‐	‐	‐	‐	‐	‐	‐	‐	‐
Christian	‐	Ref	‐	‐	Ref	‐	‐	Ref	‐
Islam	‐	1.13 (0.47–2.73)	0.78	‐	0.89 (0.41–1.96)	0.77	‐	3.84 (0.49–29.99)	0.20
*Employment status*	*1.01 (0.59)*	*‐*	*‐*	*4.34 (0.11)*	*‐*	*‐*	*3.21 (0.20)*	*‐*	*‐*
Employed by other	‐	Ref	‐	‐	Ref	‐	‐	Ref	‐
Employed by self	‐	1.29 (0.35–4.76)	0.70	‐	2.45 (0.65–9.26)	0.19	‐	2.70 (0.52–14.05)	0.23
Unemployed	‐	0.85 (0.47–1.55)	0.60	‐	0.79 (0.46–1.38)	0.41	‐	1.06 (0.40–2.80)	0.91
*Educational level*	*6.93 (0.03)*	*‐*	*‐*	*10.52 (0.01)*	*‐*	*‐*	*8.86 (0.01)*	*‐*	*‐*
Tertiary	‐	Ref	‐	‐	Ref	‐	‐	Ref	‐
Nontertiary	‐	1.10 (0.47–2.58)	0.83	‐	0.54 (0.24–1.24)	0.15	‐	0.40 (0.10–1.62)	0.19
No formal education	‐	0.62 (0.37–1.03)	0.07	‐	0.49 (0.30–0.79)	0.004	‐	0.44(0.21–0.89)	0.02
*Do you drink alcohol*	*1.37 (0.18)*	*‐*	*‐*	*0.001 (0.58)*	*‐*	*‐*	*0.92 (0.26)*	*‐*	*‐*
Yes	‐	Ref	‐	‐	Ref	‐	‐	Ref	‐
No	‐	1.95 (0.68–5.65)	0.22	‐	1.06 (0.36–3.09)	0.92	‐	1.50 (0.36–6.12)	0.58
*Comorbid conditions*	‐	‐	‐	‐	‐	‐	‐	‐	‐
Yes	0.001 (0.54)	Ref	‐	0.001 (0.54)	Ref	‐	1.70 (0.14)	Ref	‐
No	‐	1.00 (0.54–1.87)	0.99		1.14 (0.64–2.03)	‐	‐	1.69 (0.73–3.90)	0.22

Abbreviations: AOR, adjusted odds ratio; CI, confidence interval.

### 7.2 Anxiety

Marital status (AOR = 0.63, 95% CI = 0.40–1.00: *p* = 0.049) and educational level (AOR = 0.49, 95% CI = 0.30–0.79: *p* = 0.004) were associated with increased odds of reporting anxiety among participants. Participants without a regular partner were about 0.63 increased odds of experiencing anxiety during the previous week compared to those with a regular partner. Also, participants with no formal education were about 0.49 increased odds of experiencing anxiety during the past week compared to those with tertiary education (Table 3).

### 7.3 Stress

Similarly, across the total sample, only two factors showed significant bivariate associations with stress (i.e., gender and educational level), but in the logistic model, only education level showed an independent association with stress. Participants without formal education were about 0.44 increased odds of experiencing stress over the past week compared to those with tertiary education (AOR = 0.44, 95% CI = 0.21–0.89: *p* = 0.02) (Table 3).

The article "Prevalence and associations of depression, anxiety, and stress among people living with HIV: A hospital‐based analytical cross‐sectional study" was published in 2022. Journal: Health Sci Rep.

## 8 GENDER DIFFERENCES IN FACTORS ASSOCIATED WITH DEPRESSION, ANXIETY, AND STRESS

The statistical analysis was stratified according to gender to assess the bivariable and multivariable associations of the three outcomes. Interestingly, in both the bivariable and multivariable analyses, no association reached the desired threshold of statistical significance among females (Table 4). However, in males, educational level was associated with depression (AOR = 0.11, 95% CI = 0.02–0.73: *p* = 0.02) and anxiety (AOR = 0.18, 95% CI = 0.04–0.86: *p* = 0.03). Males living with HIV without formal education were about 0.11 increased odds of experiencing depression over the past week compared to those with tertiary education. Also, male participants without formal education were about 0.18 increased odds of experiencing anxiety over the past week compared to those with tertiary education (Table 5).

**Table 4:** Factors associated with depression, anxiety, and stress among females

Characteristics	Depression			Anxiety			Stress		
	*χ* ^2^ (*p*)	AOR (95% CI)	*p*	*χ* ^2^ (*p*)	AOR (95% CI)	*p*	*χ* ^2^ (*p*)	AOR (95% CI)	*p*
*Age*	*2.78 (0.25)*	*‐*	*‐*	*0.48 (0.79)*	*‐*	*‐*	*1.16 (0.56)*	*‐*	*‐*
20–39	‐	Ref	‐	‐	Ref	‐	‐	Ref	‐
40–59	‐	1.44 (0.62–3.34)	0.40	‐	1.68 (0.78–3.61)	0.185	‐	0.71 (0.23–2.22)	0.56
60–80	‐	1.75 (0.82–3.72)	0.15	‐	1.46 (0.73–2.92)	0.28	‐	0.84 (0.31–2.23)	0.72
*Marital status*	*1.09 (0.35)*	*‐*	*‐*	*2.40 (0.14)*	*‐*	*‐*	*1.05 (0.35)*	*‐*	*‐*
Currently with a regular partner	‐	Ref	‐	‐	Ref	‐	‐	Ref	‐
Currently without a regular partner	‐	0.73 (0.42–1.28)	0.28	‐	0.69 (0.41–1.16)	0.159	‐	1.84 (0.87–3.91)	0.11
*Religion*	*0.04 (>0.99)*	*‐*	*‐*	*0.24 (0.67)*	*‐*	*‐*	*3.64 (0.06)*	*‐*	*‐*
Christian	‐	Ref	‐	‐	Ref	‐	‐	Ref	‐
Islam	‐	1.14 (0.43–3.05)	0.79	‐	1.50 (0.58–3.83)	0.40	‐	‐	‐
*Employment status*	*0.94 (0.63)*	*‐*	*‐*	*2.75 (0.25)*	*‐*	*‐*	*2.75 (0.25)*	*‐*	*‐*
Employed by other	‐	Ref	‐	‐	Ref	‐	‐	Ref	‐
Employed by self	‐	1.70 (0.43–6.73)	0.45	‐	1.84 (0.45–7.50)	0.397	‐	2.96 (0.53–16.63)	0.22
Unemployed	‐	0.88 (0.44–1.74)	0.71	‐	0.60 (0.32–1.15)	0.12	‐	0.98 (0.34–2.86)	0.97
*Educational level*	*2.44 (0.30)*	*‐*	*‐*	*6.19 (0.05)*	*‐*	*‐*	*5.11 (0.08)*	*‐*	*‐*
Tertiary	‐	Ref	‐	‐	Ref	‐	‐	Ref	‐
Nontertiary	‐	0.57 (0.19–1.68)	0.31	‐	0.32 (0.11–0.88)	0.027	‐	0.30 (0.06–1.59)	0.16
No formal education	‐	0.76 (0.19–1.30)	0.31	‐	0.55 (0.33–0.93)	0.024	‐	0.48 (0.23–1.00)	0.05
*Do you drink alcohol*	*2.61 (0.18)*	*‐*	*‐*	*0.52 (0.54)*	*‐*	*‐*	*2.17 (0.15)*	*‐*	*‐*
Yes	‐	Ref	‐	‐	Ref	‐	‐	Ref	‐
No	‐	2.36 (0.67–8.32)	0.18	‐	1.39 (0.39–4.93)	0.61	‐	1.95 (0.43–8.75)	0.38
*Comorbid conditions*	*0.45 (0.63)*	*‐*	*‐*	*0.16 (0.76)*	*‐*	*‐*	*0.32 (0.65)*	*‐*	*‐*
Yes	‐	Ref	‐	‐	Ref	‐	‐	Ref	‐
No	‐	0.79 (0.40–1.58)	0.50	‐	0.94 (0.50–1.79)	0.86	‐	1.35 (0.54–3.39)	0.53

Abbreviation: CI, confidence interval.

The article "Prevalence and associations of depression, anxiety, and stress among people living with HIV: A hospital‐based analytical cross‐sectional study" was published in 2022. Journal: Health Sci Rep.

**Table 5:** Factors associated with depression, anxiety, and stress among males

Characteristics	Depression			Anxiety			Stress		
	*χ* ^2^ (*p*)	AOR (95% CI)	*p*	*χ* ^2^ (*p*)	AOR (95% CI)	*p*	*χ* ^2^ (*p*)	AOR (95% CI)	*p*
*Age*	*1.99 (0.37)*	*‐*	*‐*	*2.11 (0.35)*	*‐*	*‐*	*1.81 (0.41)*	*‐*	*‐*
20–39	‐	Ref	‐	‐	Ref	‐	‐	Ref	‐
40–59	‐	0.86 (0.13–5.68)	0.88	‐	2.58 (0.54–12.31)	0.24	‐	‐	‐
60–80	‐	0.28 (0.04–1.86)	0.19	‐	1.02 (0.25–4.14)	0.97	‐	2.88 (0.19–44.61)	0.45
*Marital status*	*0.54 (0.59)*	*‐*	*‐*	*1.78 (0.19)*	*‐*	*‐*	*0.57 (0.63)*	*‐*	*‐*
Currently with a regular partner	‐	Ref	‐	‐	Ref	‐	‐	Ref	‐
Currently without a regular partner	‐	2.26 (0.41–12.51)	0.35	‐	0.36 (0.11–1.14)	‐	‐	0.95 (0.07–13.84)	0.97
*Religion*	*0.13 (>0.99)*	*‐*	*‐*	*1.54 (0.24)*	*‐*	*‐*	*1.28 (0.32)*	*‐*	*‐*
Christian	‐	Ref	‐	‐	Ref	‐	‐	Ref	‐
Islam	‐	2.65 (0.21–32.98)	0.45	‐	0.36 (0.06–2.11)	0.25	‐	0.42 (0.02–8.36)	0.57
*Employment status*	*0.91 (0.64)*	*‐*	*‐*	*2.38 (0.30)*	*‐*	*‐*	*0.07 (0.97)*	*‐*	*‐*
Employed by other	‐	Ref	‐	‐	Ref	‐	‐	Ref	‐
Employed by self	‐	‐	‐	‐	‐	‐	‐	‐	‐
Unemployed	‐	1.08 (0.20–5.93)	‐	‐	2.26 (0.55–9.29)	‐	‐	0.40 (0.02–9.51)	0.57
*Educational level*	*16.27 (<0.001)*	*‐*	*‐*	*9.60 (0.01)*	*‐*	*‐*	*1.67 (0.43)*	*‐*	*‐*
Tertiary	‐	Ref	‐		Ref	‐	‐	Ref	‐
Nontertiary	‐	2.77 (0.35–21.78)	0.93	‐	1.07 (0.16–7.10)	0.94	‐	0.31 (0.01–11.60)	0.53
No formal education	‐	0.11 (0.02–0.73)	0.02	‐	0.18 (0.04–0.86)	0.03	‐	0.11 (0.00–2.90)	0.18
*Do you drink alcohol*	*0.003 (>0.99)*	*‐*	*‐*	*0.61 (0.66)*	*‐*	*‐*	*0.28 (1.00)*	*‐*	*‐*
Yes	‐	Ref	‐	‐	Ref	‐	‐	Ref	‐
No	‐	1.91 (0.10–37.10)	0.67	‐	0.64 (0.05–7.57)	0.72	‐	‐	‐
*Comorbid conditions*	*1.82 (0.23)*	*‐*	*‐*	*0.40 (0.53)*	*‐*	*‐*	*4.82 (0.09)*	*‐*	*‐*
Yes	‐	Ref	‐	‐	Ref	‐	‐	Ref	‐
No	‐	5.51 (0.76–39.94)	0.09	‐	2.28 (0.45–11.47)	0.32	‐	10.91 (0.63–188.49)	0.10

Abbreviation: CI, confidence interval.

## 9 DISCUSSION

This study assessed the prevalence estimates of depression, anxiety, and stress and identified some of the socio‐demographic factors associated with these mental health challenges among PLHIV presenting to a teaching hospital in Ghana. Key findings indicate relatively high prevalence estimates of depression, anxiety, and stress. Approximately, 4 out of 10 PLHIV experienced depression, about 1 out of 5 reported anxieties, and 1 out of 10 self‐reported stress during the previous week. Relative to estimates reported by previous studies from high‐income countries, the estimates in the current study appear higher.^16^, ^17^ In the United Kingdom, the prevalence estimates of depression and anxiety among people living with HIV in the past 2 weeks were 19.8% and 13.1%, respectively.^16^

The article "Prevalence and associations of depression, anxiety, and stress among people living with HIV: A hospital‐based analytical cross‐sectional study" was published in 2022. Journal: Health Sci Rep.

Interestingly, it does appear that the estimates of the current study are comparable to estimates from other low‐ and middle‐income countries. For example, a cross‐sectional study in South Ethiopia using the hospital anxiety and depression scale indicated 32.0% and 34.4% prevalence of depression and anxiety, respectively among PLHIV.^4^ Similarly, a study in India using DASS‐21 reported that 50% PLHIV suffered from depression.^3^ Although the prevalence estimates of depression and anxiety (as reported by the current and previous studies) are high, the values still differ, particularly, when the estimates are viewed in actual counts/values. The prevalence estimates of depression, anxiety, and stress among PLHIV have been observed to differ worldwide.^16^, ^17^, ^18^, ^19^, ^20^, ^21^, ^22^ Differences in the estimates have been attributed to different settings and methodological approaches used by available studies. In addition, cultural difference in response to surveys on mental health issues and social desirability bias due to social or self‐stigma might have contributed more to the similarities (than differences) in the estimates across low‐ and middle‐income countries.

The current study has also shown that females are more likely than males to report depression, anxiety, and stress. This evidence is consistent with findings from similar studies.^4^, ^19^, ^23^ Generally, this finding is not surprising for the reason that females tend to experience and report more internalizing problems than males.^24^ This study's findings further indicate that, a vast majority of PLHIV do not drink alcohol. It appears that, the estimates from this study are not consistent with findings of similar studies which indicate a high incidence of alcohol use among PLHIV.^28^, ^29^, ^30^ Maladaptive means of coping may lead to an increase in the use of alcohol among PLHIV and may impact their health negatively.^29^, ^30^ The low consumption of alcohol among PLHIV in this current study, may be associated with the use an adaptive coping strategy. PLHIV require a great deal of social and emotional support to help them deal with the psychosocial burden of living with the virus.^25^ However, within the socio‐cultural setup of Ghana, sexually transmitted diseases are highly stigmatized and gender inequality is still pervasive; women continue to experience inequality, lower social status, and increased vulnerability to discrimination and various forms of abuse.^25^ In these circumstances, women living with HIV are more likely (than men) to experience social adversities, social ostracism and isolation, and an inability to attract meaningful social support, thereby increasing their vulnerability to negative mental health outcomes such as loneliness, depression, and anxiety.

The article "Prevalence and associations of depression, anxiety, and stress among people living with HIV: A hospital‐based analytical cross‐sectional study" was published in 2022. Journal: Health Sci Rep.

The study findings suggest also that PLHIV without a regular partner are more likely to report anxiety compared to those with a regular partner. A cross‐sectional study in Zambia also found high prevalence of depression among unmarried, widowed, and divorced women.^19^ People who are in less stressful marriages may be less vulnerable to mental health challenges.^26^ Although marriage may not necessarily militate against the onset of mental illness in partners, meaningful spousal support may promote resilience and could present as a potential protective factor against mental health challenges among persons in marital relationships.^27^ For PLHIV, having a supportive spouse is critical to promoting resilience in the face of mental health challenges.^28^

The key finding that PLHIV without formal education (compared to those with tertiary education) are at increased odds of experiencing anxiety and stress is worth some comments. This evidence could be pointing to an outcome of the functional health literacy that PLHIV with formal/tertiary education must have received by virtue of having had formal classroom education. HIV/AIDS literacy remains a detailed part of the health education curriculum from basic schools through tertiary educational institutions in Ghana.^29^ The implication is that, on the one hand, PLHIV who have had some formal education are more likely to hold educated beliefs about the virus and to draw on their acquired classroom knowledge and HIV literacy contents to inform their health behavior choices and coping strategies. PLHIV who have had no formal education, on the other hand, may struggle (possibly without success) in their attempt to generate alternative courses of action, as they lack educated knowledge about the virus and how to live with it. While further research is needed to clarify this supposed association between functional health literacy and reduced negative mental health outcomes in PLHIV who have formal/tertiary education background, perhaps, this finding also underscores a need to consider designing a functional health literacy program targeted at PLHIV without formal education who present to antiretroviral clinics in Ghana.

The article "Prevalence and associations of depression, anxiety, and stress among people living with HIV: A hospital‐based analytical cross‐sectional study" was published in 2022. Journal: Health Sci Rep.

The strengths of this study include the use of a standardized measure to assess the prevalence estimates of depression, anxiety, and stress. The application of standardized measures strengthens a study's contributions to relatively valid estimates of outcomes. Also, the sample size used for this study was representative of the population of PLHIV presenting to the Cape Coast Teaching Hospital. However, this study had some limitations. The study was a cross‐sectional survey, therefore did not establish cause and effect relationship between associated factors and outcomes (depression, anxiety, and stress). Notably, this study failed to measure antiretroviral adherence/medical adherence, number of years lived with HIV/illness duration, and social adversities experienced due to HIV, while most of the included “exposure variables” were socio‐demographic factors which in themselves may not necessarily be modifiable (risk or protective) factors related to the outcomes. It is important to consider this point in designing related studies in the future, particularly, in Ghana and other sub‐Saharan contexts.

## 10 CONCLUSIONS

The levels of depression, anxiety, and stress are high among PLHIV in Ghana, and females report disproportionately higher levels. However, the effects of mental health problems among PLHIV are often underestimated, and this is more serious in a resource‐constrained country like Ghana and its sub‐Saharan context. The mental health care system in Ghana is grossly underfunded and provides little by way of screening and treatment for PLHIV. It is important for the managers of the healthcare system to integrate mental health assessment and management in the HIV care services. There is a need to build the capacity of health care workers to offer differentiated service delivery based on the mental health care needs of PLHIV. Primary care providers should be trained to provide mental health care services such as mental health assessment, counseling, and psychosocial support to PLHIV.

## AUTHOR CONTRIBUTIONS

*Sampson Opoku Agyemang*: conceptualization, data curation, formal analysis, methodology, project administration, writing—original draft, writing—review & editing. *Jerry Ninonni*: conceptualization, data curation, methodology, project administration, supervision, writing—original draft, writing—review & editing. *Lydia Bennin*: conceptualization, data curation, methodology, project administration, writing—review & editing. *Elizabeth Agyare*: data curation, project administration, writing—review & editing. *Leveana Gyimah*: project administration, writing—review & editing. *Kafui Senya*: project administration, writing—review & editing. *Emmanuel Birikorang*: formal analysis, methodology, writing—review & editing. *Emmanuel Nii‐Boye Quarshie*: formal analysis, methodology; supervision, writing—original draft, writing—review & editing. *Nyonuku Akosua Baddoo*: methodology, project administration, supervision, writing—review & editing. *Stephen Ayisi Addo*: conceptualization, project administration, writing—review & editing. *Dorcas Obiri‐Yeboah*: conceptualization, formal analysis, methodology, project administration, supervision, writing—original draft, writing—review & editing. All authors have read and approved the final version of the manuscript. Corresponding author had full access to all of the data in this study and takes complete responsibility for the integrity of the data and the accuracy of the data analysis.

The article "Prevalence and associations of depression, anxiety, and stress among people living with HIV: A hospital‐based analytical cross‐sectional study" was published in 2022. Journal: Health Sci Rep.

## CONFLICT OF INTEREST

The authors declare no conflict of interest.

## ETHICS STATEMENT

This study was performed in accordance with the Helsinki Declaration and approved by the Ethics Review Committee of Cape Coast Teaching Hospital, Ghana (reference: CCTHERC/EC/2021/028). The purpose of the study, anonymity, voluntary participation, and confidentiality of the information were explained to participants to seek their written consent. Participants could withdraw from the study at any point without any adverse effect.

## TRANSPARENCY STATEMENT

Sampson Opoku Agyemang affirms that this manuscript is an honest, accurate, and transparent account of the study being reported; that no important aspects of the study have been omitted.

## Data Availability

The authors confirm that the data supporting the findings of this study are available within the article. However, the data are available from the corresponding author upon reasonable request.
